RETRACTED

# Probiotics from Dairy Products on Intestinal Barrier Function Using Caco-2 Cells under Microscope

**DOI:** 10.1155/2022/6293095

**Published:** 2022-08-08

**Authors:** Peilin Yao, Jiaxuan Jiang, Zhenyang Kong

**Affiliations:** School of Biological and Food Engineering, Suzhou University, Suzhou, 234000 Anhui, China

## Abstract

With the continuous improvement of human living standards, people's demand for health has become an important international research hotspot. In recent years, 41.3% of the total incidence of multiple organ failure (MOF) caused by dysfunction of the intestinal screen was found every year. The mortality rate is 62%, which is more than twice that of developed countries. This paper is aimed at observing the microscopic effects of probiotics derived from dairy products using Caco-2 cells on intestinal barrier function. Based on the above background, the purpose of this study was to construct a Caco-2 cell model under microscope to study the effect of probiotics on intestinal barrier function. This study first describes the background knowledge of the integration of modern microscope technology and medical field and the correlation between them. The results showed that the relative adhesion rates of Lactobacillus bulgaricus, Lactobacillus acidophilus, and Streptococcus thermophilus were 4.67 ± 0.07%, 11.53 ± 0.06%, and 18.31 ± 0.08%, respectively, which were lower than those in the normal group. The production of antibacterial substances can inhibit intestinal pathogens and adjust the balance of intestinal flora.

## 1. Introduction

With the continuous development of the global economy, people's life rhythm is also accelerated. People continue to pursue high efficiency after work. Takeout and fast food have become staple food, which leads to many gastrointestinal problems. Moreover, this situation is developing to a younger age, so it has attracted the attention of modern people. Since people began to pay attention to gastrointestinal problems, most people's understanding of intestinal function may lie in the digestion and absorption of daily nutrients, and the monitoring indicators and treatment of intestinal function only stay in the aspects of digestion and absorption of nutrients and parenteral nutrition (PN) [1]. The concept and research of intestinal comprehensive function have not been paid enough attention. With the continuous exploration of clinical medicine and the cognition of PN deficiency in recent ten years, it has been found that the damage of intestinal barrier function is the important factor of intestinal bacterial translocation and systemic inflammatory response syndrome (SIRS), which is also the main cause of multiple organ dysfunction syndrome (MODS) and multiple system organ failure (MSOF) [2]. Based on the information collected, people began to regard intestinal barrier function as a criterion to judge the prognosis of critically ill patients. Some even call the gut “the center of the problem of organ production when the body is stressed.” However, the etiology, diagnosis, prevention, and treatment measures are not perfect, and more in-depth research should be carried out. With the emergence and rapid development of microscope technology, new tools have appeared in the study of intestinal barrier function in medical field, and the treatment of intestinal barrier function has also made a historic leap [3].

RETRACTED

Zhou selected 180 IBD patients as research objects to study the protection of intestinal barrier. To evaluate the intestinal barrier injury, diamine oxidase (DAO), D-lactic acid (d-la), and bacterial lipopolysaccharide (BET) were selected to evaluate the intestinal barrier injury. Combined with the recommendations of gastrointestinal dysfunction classification proposed by the European intensive care medicine association (ESICM) annual meeting in 2012, the clinical classification of acute gastrointestinal dysfunction (AGI) was carried out for IBD patients, which provided the basis for barrier function damage of IBD and provided reference for the formulation of treatment strategies and the preevaluation [4]. Hua et al. studied the role of fatty acid-binding protein (iFABP) as a sample of intestinal barrier function in the changes of intestinal flora and found that the integrity of intestinal mucosal barrier in obese patients can be damaged by dietary fat, resulting in increased intestinal permeability. However, obesity induced by high-fat diet is characterized by physiological disorder, insulin resistance, and systemic inflammatory response. In this case, blood iFABP should not be used as a marker of intestinal mucosal barrier function and mild chronic inflammation [5]. Although the current research results are relatively rich, there are still deficiencies, mainly reflected in the limitations of the current methods for the examination of intestinal barrier function.

As people pay more and more attention to the health problems, the safety of probiotics has been paid more and more attention. The emergence of probiotics in dairy products has attracted much attention in recent years, because it is a kind of bacteria beneficial to human body. It can be directly used as an auxiliary additive in daily food without any treatment and can be used to protect the balance between intestinal flora. But the source of probiotic strains, its safety, effectiveness, and controllability should be carefully examined. Gao and other experts have found that the growth rate of probiotic milk drinks is very fast, reaching an average annual growth rate of 27%, and this trend will remain unchanged in the next three years [6]. This data strongly shows that probiotic dairy products are sought after by consumers because of their high nutritional value and unique health functions. However, the production technology of probiotics is relatively backward. Therefore, in the future development of probiotic products, we should further study the mechanism of strains, so as to further screen strains with specific functions that can meet the needs of different age groups [7]. Song selected stinky tofu and Sufu from Changchun and two different rural areas in Heilongjiang Province to collect fermented food glutinous flour and homemade chili sauce samples and expected to screen lactic acid bacteria strains with good probiotic function. Lactic acid bacteria can produce acid in the process of fermentation. Most of the cells are Gram-positive bacteria, with spherical and rod-shaped cell morphology. At present, the common method is based on the phenotypic characteristics and 16SrRNA gene sequence. It cannot distinguish the bacteria strains of the same genus obviously, and sometimes the strains of different genera are different [8]. The data of these studies are not complete, and the experimental conclusions are still open to question, so they cannot be widely used in the public field. Nowadays, probiotics in dairy products have been widely used. There are 392 kinds of probiotics in dairy products, but there are only more than 30 kinds of probiotics put into production, and the utilization rate of strains is less than 7%. Therefore, screening suitable lactic acid bacteria is the focus of current research.

RETRACTED

In order to observe the effect of dairy probiotics on intestinal barrier function, Caco-2 cells were used to study the effect of dairy probiotics on intestinal barrier function.

## 2. Intestinal Barrier Function of Probiotics in Dairy Products by Caco-2 Cells

### 2.1. Microscope-Assisted Technology

Microscope research has been going on for a long time. As the most common three kinds of microscopic imaging technology, bright field, dark field, and phase microscopic imaging have also achieved different degrees of development over the years [9]. Compared with the other two techniques, it is easier to realize the bright field microscopic imaging technology. And because the price of using the technology is more civilian, so the scope of use of the technology is also relatively wide. However, the effect of this technology on the contrast of imaging results is relatively poor. In particular, in the use of some transparent samples, we cannot get the results we need. Therefore, many experts have proposed many improvement measures, such as dyeing the observed samples or improving the imaging contrast through defocusing [10]. And we can get a clear image of the sample with large scattering angle. In the early days, the ring electron microscope was often used to observe the dark field. The principle is to use ring detector to collect scattered electrons in the sample to realize imaging. In recent years, based on the imaging characteristics of dark field microscopy, it has been widely used in the field of electron microscopy, thus further combining dark field imaging with traditional digital holography; this method is a supplement to bright field microscopy imaging. However, the traditional phase contrast microscope technology is suitable for materials with weak absorption, small attenuation of X-ray and light, and large phase transition. In the past few decades, many imaging methods based on phase information have been developed, including traditional phase contrast microscopy and intensity transfer function (tie: transport intensity equation and digital holography), white light double fractional tomography (wbd-X-ray tomography: 1 WDT, optical coherence tomography (OCT), diffraction phase microscopy (DPM): diffraction). With the passage of time, more and more new methods have been published in high impact journals, which shows that this technology field is active.

### 2.2. Caco-2 Cell Model

Caco-2 cells are derived from human colon cancer cells. This kind of cells can automatically differentiate into intestinal cell like cells in the general culture environment, which can be used as a model of small intestinal epithelial cells to study the transmembrane transport of drugs [11]. Because the use effect of drugs through Caco-2 cell model is more conducive to experts' research than the effect of oral drug absorption, the research of drug transport in the intestinal tract has reached a new height in the field of cells. In addition, because of the good reproducibility of Caco-2 cell model, it is often used in studying the relationship between drug structure, absorption, and transport, the influence of dosage forms and excipients on absorption, the mechanism of oral drug absorption and transport, and the optimal pH value of drug absorption in the small intestine. The formation of the Caco-2 cell model is different due to different culture conditions. The methods of evaluating Caco-2 cell model are as follows: observing the morphology of Caco-2 cells with electron microscope or optical inverted microscope, measuring AKP activity of brush border cells of small intestine, measuring transmembrane resistance; measuring the permeability of Caco-2 cells with fluorescent or radioactive markers such as mannitol and fluorescein horseradish peroxidase (HRP), and determining the permeability of Caco-2 cells with phenolphthalein [12]. In this experiment, Caco-2 cells crawl into thin slices. After cell differentiation, Caco-2 cells were cocultured with Lactobacillus bulgaricus, Lactobacillus acidophilus, and Streptococcus thermophilus for 24 h. The Caco-2 cells labeled with *β*-tubulin were labeled by immunofluorescence method, and the images were collected by a confocal microscope for processing [13].

RETRACTED

### 2.3. Probiotics in Dairy Products

As early as ancient times, people's daily diet already contained lactic acid fermented food. In general, the most important probiotics include Lactobacillus and Bifidobacterium. Probiotics mainly come from natural fermented dairy products and are obtained by artificial screening. It is defined as a group of living microorganisms that produce one or more functional health benefits to the host through adequate intake. With the development of probiotics research, the probiotic function of probiotics has been gradually developed and utilized [14, 15].

### 2.4. Intestinal Barrier Function

The intestinal tract is the organ with the most bacteria in human body, which contains about 1013-1014 kinds of bacteria. Microorganisms in the gut play a dual role in intestinal barrier function. From one point of view, as bacteria, it has a certain degree of harm, and at the same time, there are some hidden dangers to the intestinal barrier function; from another point of view, the microorganisms in the intestinal tract can provide some of the nutrients needed by the cells in the intestinal tract, ensure the microecological balance of the intestinal tract, make the immune system of the intestinal tract in a startup state, and form the intestinal barrier function one link. The pathogenic bacteria in the intestine and the ability of the bacteria to destroy the intestinal barrier function can directly destroy the tight junction protein, leading to the decline of intestinal cell resistance. For example, enterohemorrhagic Escherichia coli, another mechanism, is indirectly leading to tight junction rupture [16, 17], such as coliform injury caused by intestinal disease. It has been found that enteropathogenic Escherichia coli secretes an espf protein through its type I secretion system. In addition, pathogenic Escherichia coli can also produce some toxins, such as Helicobacter pylori toxin, Clostridium difficile toxin A and B, and Pseudomonas aeruginosa exotoxin. These toxins can affect the permeability of intestinal epithelium without causing structural changes of tight junction. In addition, botulinum and Listeria can cause intestinal barrier dysfunction by regulating actin cytoskeleton. Amoeba and other microorganisms can produce amoeba cysteine protease, which stimulates NFkB transcription factor of human intestinal epithelial cells. Through the release of IL-1*β*, it can cause intestinal inflammation and damage intestinal epithelial cells. Some intestinal parasites also protect the gut barrier. These intestinal symbionts are mainly obligate anaerobes, including Lactobacillus and Bifidobacterium. These microorganisms have ecological stability and can resist and repel the invasion of exogenous pathogens and intestinal mucosal cells. At the same time, the symbiotic bacteria on the surface of intestinal mucosa can directly regulate inflammatory transcription factors such as nfrb and regulate the intestinal anti-infection ability. It has been found that some symbionts can regulate the expression of some genes that play an important role in intestinal barrier function, such as nutrient absorption, intestinal mucosal barrier structure formation, heterogeneous biochemical metabolism, angiogenesis, and intestinal epithelial cell maturation and differentiation. The chemical substances secreted by intestinal bacteria and intestinal mucus are composed of chemical substances secreted by intestinal bacteria. IgM and other antibodies secreted by intestinal epithelial cells and submucosal lymphoid tissue constitute the mucosal barrier; the colonization resistance and aggregation of normal intestinal symbionts to pathogenic bacteria constitute biological screening [18]. Any part of the above injury may lead to the impairment of intestinal barrier function.

RETRACTED

## 3. Experimental Study on Intestinal Barrier Function of Probiotics

### 3.1. Experimental Instruments and Equipment

The equipment needed are carbon dioxide incubator, digital display constant temperature water bath pot, ordinary optical microscope, analytical balance, inverted microscope, electric blast drying oven, ultraclean workbench, table-type constant temperature oscillator, enzyme label analyzer, centrifuge, biochemical incubator, ordinary refrigerator, seat type electrothermal pressure steam sterilizer, liquid nitrogen biological container, electronic balance, laboratory pH meter, 96-holes culture plate, 0.22 *μ*m microporous membrane, blood cell counting plate, micropipette, and other chemical instruments: alcohol lamp, 75% alcohol cotton, etc.

### 3.2. Experimental Sample Cells and Strains

Caco-2 cells (human colon cancer cells), bulgaricus, Streptococcus thermophilus, Lactobacillus acidophilus were used.

### 3.3. Experimental Methods

Caco-2 cells were made into cell suspension and divided into equal groups. Caco-2 cells were counted by blood cell counting method: a special cover glass was placed in the center of the cell counting board, and the mixed cell suspension was absorbed by a micro pipette and discharged from the pit of the counting plate under the cover glass until the cover glass was filled with liquid. The total number of cells in the four corners of the square was counted under the inverted microscope. The remaining cell suspension was placed in the refrigerator for standby, and different probiotics were added for culture. The recovery of probiotics is to take the lyophilized powder from the ultralow temperature refrigerator, balance at 40°C for 10 minutes, then loosen the plastic tube on the super clean table, take out the sealed ampoule tube, wipe it with alcohol cotton ball, heat the top of the ampoule tube with alcohol lamp flame, and then drop a cup of sterile distilled water. At this time, obvious cracks appeared on the top of ampoule tube. Use tweezers to tap the crack, knock open the ampoule tube, add a small amount of sterile normal saline, gently shake to dissolve freeze-dried bacteria into suspension, take a certain amount of bacterial liquid into the sterilized MRS broth medium, put it into the biochemical incubator, activate the medium at 37°C, and the inoculation rate is 3%. After three generations of culture, the bacterial activity reached the experimental requirements. Take the bacterial suspension smear, observe the colony morphology under the microscope, and take appropriate amount of probiotics smear. Lactobacillus bulgaricus, Lactobacillus acidophilus, and Streptococcus thermophilus were inoculated in a test tube containing 5 ml MRS fresh broth medium. The absorbance values were measured at 4 h, 8 h, 12 h, 16 h, 20 h, 24 h, 28 h, and 32 h, respectively. The concentration of Caco-2 cell suspension was adjusted to 1.5 × 10^5^ cells/ml, and 100 *μ*l was added into each well of a 96-well plate. After 24 hours, probiotics (Lactobacillus bulgaricus, Lactobacillus acidophilus, and Streptococcus thermophilus) were cultured at 5% CO_2_ and 37°C. Each group has 3 wells and blank control group. After 24 h, the supernatant was discarded, washed with sterile PBS for 3 times, MTT was added and incubated for 4 h. The supernatant was discarded and added with DMSO, 150 *μ*l per well. The OD value of absorbance was determined at 490 nm. Finally, the experimental data are collected.

## 4. Analysis of Intestinal Barrier Function of Probiotics in Dairy Products

### 4.1. Adhesion Inhibition Method

The antagonistic effects of three probiotics on Caco-2 cell adhesion are shown in Table 1.

RETRACTED

The results showed that the colonization of host cells and the formation of membrane microflora in competitive sites could effectively inhibit the growth of pathogenic bacteria or opportunistic pathogens, maintain the inherent intestinal flora, and ensure the secretion of lysozyme and proteolytic enzyme, so as to control the infection. The interaction between microorganism and host intestine is the premise of the existence of intestinal microorganism [19].

### 4.2. Toxicity Analysis of Three Common Probiotics on Caco-2 Cytokines

The intestinal tract is not only the place where the human body digests and absorbs but also plays the function of immune organs. The surface area of intestinal mucosa is very large, and hundreds of millions of microorganisms coexist with it. Therefore, the intestinal mucosa constitutes the mucosal immune system and plays the role of intestinal barrier. Intestinal epithelial cells participate in the innate immunity of intestinal mucosa and play an important role in the invasion of pathogenic microorganisms. They secrete cytokines to carry out a series of immune responses to maintain the stability of intestinal environment and human health. The Caco-2 cell model was used to study whether Lactobacillus bulgaricus, Lactobacillus acidophilus, and Streptococcus thermophilus could cause intestinal barrier dysfunction. The results are shown in Figure 1.

It can be seen from the figure that the three probiotics did not cause abnormal secretion of cytokines. Different bacterial concentrations have different effects on Caco-2 cytokines.

### 4.3. Analysis of the Influence of Three Common Probiotics on Caco-2 Cell Monolayer Model

Phenol red permeation test is a means to detect the integrity of the monolayer, and the formation of the integrity of the Caco-2 monolayer can be observed while measuring the permeation amount of phenol red. The transmembrane flux of monolayer was measured by phenol red transmission rate method. The standard curve of phenol red is shown in Figure 2.

In this study (Figure 3**)**, the Caco-2 cell monolayer model was used to coculture probiotics with high concentration. After fixation, embedding, and ultrathin section, the tight junction structure was observed under a transmission electron microscope.

### 4.4. Effects of Three Common Probiotics on Caco-2 Cytoskeleton

*β*-Tubulin (*β*-tubulin) is an important component of cytoskeleton. After being treated with 10^8^ CFU/ml Lactobacillus bulgaricus, Lactobacillus acidophilus, and Streptococcus thermophilus for 24 hours, the *β*-tubulin of Caco-2 cells was labeled by immunofluorescence method, and the green light of *β*-tubulin was observed under laser confocal microscope. Immunofluorescence method is a method that combines immunological methods (antigen-antibody specific binding) with fluorescent labeling technology to study the distribution of specific protein antigens in cells. The specific results are shown in Table 2.

RETRACTED

After differentiation, Caco-2 cells were cocultured with 10^8^ CFU/ml Lactobacillus bulgaricus, Lactobacillus acidophilus, and Streptococcus thermophilus, respectively, for 24 h. The *β*-tubulin-labeled Caco-2 cells were detected by immunofluorescence method, and the images were collected and processed by a confocal microscope. The results showed that the fluorescence intensity of *β*-tubulin in Caco-2 cells cocultured with probiotics and Caco-2 cells had no significant difference, indicating that Lactobacillus bulgaricus, Lactobacillus acidophilus, and Streptococcus thermophilus had no effect on *β*-tubulin of Caco-2 cells.

### 4.5. Results of Cell Bypass Mannitol Permeability and Intestinal Epithelial Cell Transmembrane Resistance after Different Probiotics Treatment

The results of the paracellular mannitol permeability and intestinal epithelial cell transmembrane resistance after different probiotic treatments are shown in Figure 4.

As can be seen from the figure, these studies suggest that infection can destroy the intestinal barrier function and cause bacterial or toxin translocation. Probiotics can promote the recovery of intestinal epithelial cell junction and protect intestinal mechanical barrier.

## 5. Conclusions

In this study, the potential probiotics of Lactobacillus plantarum in traditional dairy products were systematically discussed through in vitro evaluation test, and some Lactobacillus plantarum had potential probiotic potential for the first time. The results showed that the growth inhibition ability of the tested strains was different, but most of them had extensive inhibitory effect on the growth of selected pathogens. If the antibacterial activity can be expressed in vivo, it seems to be beneficial to maintain the balance of normal intestinal flora. At the same time, the test also showed that the antibacterial effect of the experimental strains against nonpathogenic bacteria was weak.

In this paper, three probiotics (Lactobacillus bulgaricus) were used to study the effect of probiotics (2) on colon cancer cells in vitro. In order to investigate the potential safety of probiotics in dairy products and provide technical support for the screening of probiotics strains and the development of probiotics in dairy products in China, the effects of different concentration and combination of strains on the proliferation of Caco-2 cells were investigated. The tight junction structure was observed under the microscope, and the distribution of cytoskeleton protein *β*-tubulin was observed under the confocal laser. The cells used in this study are too single, which is not conducive to the widespread popularization of the study, so it is recommended to use several kinds of cells.

RETRACTED

## Figures and Tables

**Figure 1:** Effects of different probiotics on Caco-2 cytokines.

**Figure 2:** Phenol red standard curve.

**Figure 3:** The effect of different probiotics on the transmission rate of phenol red.

**Figure 4:** Cumulative permeability of mannitol.

**Table 1:** Antagonistic effects of three probiotics on adhesion of Caco-2 cells.

Grouping	Relative adhesion rate (mean ± SD)%	Colony count (mean ± SD)
Control group	100 ± 0.00	1.2 × 10^6^ ± 1.7 × 10^5^
Bulgaricus group	4.67 ± 0.07	0.47 × 10^5^ ± 0.6 × 10^4^
Streptococcus thermophilus group	11.53 ± 0.06	1.31 × 10^5^ ± 1.1 × 10^4^
Lactobacillus acidophilus group	18.31 ± 0.08	1.83 × 10^5^ ± 1.6 × 10^4^

**Table 2:** Effects of different probiotics on cytoskeleton *β*-tubulin of Caco-2 cells.

	Bulgarian group	Lactobacillus acidophilus	Streptococcus thermophilus	Control group
Relative strength	9	9	8	9

## Data Availability

No data were used to support this study.
